# Does the discrepancy between implicit and explicit attitudes moderate the relationships between explicit attitude and (intention to) being physically active?

**DOI:** 10.1186/s40359-019-0322-z

**Published:** 2019-08-07

**Authors:** Carolin Muschalik, Iman Elfeddali, Math J. J. M. Candel, Rik Crutzen, Hein de Vries

**Affiliations:** 1 Department of Health Promotion, Care and Public Health Research Institute (Caphri), Maastricht University, P.O. Box 616, 6200 MD Maastricht, The Netherlands; 2 GGz Breburg, Academic Department of Specialized Mental Health Care, P.O. Box 770, 5000 AT Tilburg, The Netherlands; 3 Tranzo - Scientific Center for Care and Welfare, Tilburg University, P.O. Box 770, 5000 AT Tilburg, The Netherlands; 4 Department of Methodology and Statistics, Care and Pubic Health Research Institute (Caphri), Maastricht University, P.O. Box 616, 6200 MD Maastricht, The Netherlands

**Keywords:** Implicit attitude, Explicit attitude, Implicit-explicit discrepancy, Intention, Physical activity

## Abstract

**Background:**

Explicit attitudes as well as implicit attitudes have been shown to be associated with physical activity (PA). These two types of attitudes can, however, be discrepant towards the same object or behavior. This study investigated whether there is a discrepancy between explicit and implicit attitudes (IED) regarding physical activity (PA), and whether IED moderates the relationship between explicit attitude and PA, and explicit attitude and PA intention.

**Methods:**

At baseline (T0) and one (T1) and three months (T2) thereafter, students’ (*N* = 340) PA levels, intention, explicit attitudes, further PA determinants, e.g. self-efficacy, were assessed. Implicit attitudes towards PA were assessed by means of a tailored Single-Category Implicit Association task.

**Results:**

IED was present but weak. Multiple hierarchical regressions revealed that IED did not moderate the relationship between explicit attitudes and PA or intention. Yet, IED was negatively associated with T0-PA and T1-PA.

**Conclusion:**

The study revealed the important insight that IED is detrimental for PA. Interventions targeting attitudes to increase PA, should ensure that implicit and explicit attitudes regarding PA are concordant.

Explicit attitudes are a key construct in many behavioral theories and a relevant determinant across a wide range of health behaviors [1–5]. They are defined as conscious attitudes that are formed deliberately, which implies that people can self-report on their explicit attitudes (e.g. in a questionnaire). Explicit attitudes are composed of instrumental and affective components [6, 7]. Whereas the instrumental component refers to anticipated positive or negative consequences that would result from performing a behavior, the experiential component is understood as emotion-laden judgments about a behavior. In recent decades, implicit attitudes have gained increased attention to serve as additional constructs for predicting and explaining health behaviors. They can be understood as mental associations between a concept (e.g. physical activity) and a favorable or unfavorable evaluation (e.g. positive or negative) [8] to which people do not have or sometimes do not want to have conscious access (Rydell & McConnell, 2006). The strength of these associations manifests automatically into behavioral tendencies without the need for reflection. This has been demonstrated for a variety of behaviors [for example] [9, 10]. To capture these associations, mostly reaction time paradigms are used. An example is the Implicit Association Test (IAT) in which participants have to sort words or pictures to given categories as quickly as possible [11]. The underlying idea is that the stronger a negative or positive association in mind, the quicker is a person with categorizing the stimuli to the respective category. Based on that, inferences about the person’s implicit attitude towards a specific object or behavior can be drawn. Dual-process models, such as the Reflective-Impulsive Model [12] or the Associative Propositional Evaluation Model (APE) [13] depict that both explicit and implicit attitudes can be associated with behavior.

The relationship between behavior on the one hand, and implicit and explicit attitudes on the other hand, may however differ for different types of behaviors. For example, implicit attitudes are more strongly associated with spontaneous behavior and explicit attitudes with deliberate behavior [14–16]. For certain behaviors, such as voting behavior [17] or physical activity [9, 18], the two attitude-types can also have a joint effect. Furthermore, it has been shown that implicit and explicit attitudes towards one behavior do not always coincide: they can be discrepant, meaning that the explicit attitude towards a behavior is for example negative whereas the implicit attitude is positive or vice versa. This is called the implicit-explicit discrepancy (IED). In the study at hand, the effect of IED on the relationship between explicit attitude and behavior and explicit attitude and intention is investigated.

The existence of IED has been demonstrated in several studies [19–21] and different factors have been discussed as possible sources for IED, such as self-presentational concerns (e.g. explicit measures are more likely to diverge from an implicit measure when self-presentational concerns are high) [22, 23], preference for consistency (e.g. individuals with a stronger distinct motivation to seek congruence between their cognitions show lower IED compared to people with a less distinct preference for consistency) [24], or methodological factors such as the consistency of the content assessed by the implicit and explicit measure (e.g. lower IED when the content of the measures is consistent) [25]. The APE also put forward theoretical assumptions about the existence of IED [13]. According to the APE, there exist two independent systems of reasoning. First, the slow-learning system, which operates by using interconnected associations in memory that are based on contiguity and similarity. Hence, learning takes place by the establishment of associations in memory that are formed slowly over time. Implicit attitudes are attributed to the slow-learning system. The second system, the fast-learning system, is assumed to rely on logic at a higher level of cognitive processing, which fits with the conceptualization of explicit attitudes and indicates that people can have control over the expression of their explicit attitudes and that they can be changed more quickly [26]. Hence, it is possible that a change in explicit attitude happens faster than a change in a person’s implicit attitude, thereby resulting in dissonance between implicit and explicit attitudes [21]. Also, as implicit and explicit attitudes are ascribed to two different systems, they might be influenced by different processes. For example, in one study explicit attitudes were changed by means of verbally presented behavioral information whereas implicit attitudes were changed by subliminally presented primes [27]. When only one type of change method is used, asymmetric changes can occur [21, 28] (e.g. when only one type of attitude is changed by means of a specific method that leaves the other attitude unaddressed), resulting in a dissonance between attitudes.

Although dissonance has repeatedly been demonstrated, only a few studies assessed the effect of IED on *behavior* [19, 20, 29–31]. Concerning this relationship, inconsistent patterns were found. For example, in a study on the consequence of discrepant attitudes on information processing Briñol et al. [19] found that people with a greater discrepancy between their implicitly and explicitly measured self-dimensions, e.g. self-esteem, engaged in a more thorough elaboration of attitude-relevant information (but not of attitude-irrelevant information) than people with consistent self-dimensions. Also Rydell and colleagues [29] demonstrated that diverging implicit and explicit attitudes towards a specific target person resulted in dissonance and in additional information processing about that person. The authors of both studies assumed that the higher information processing was a result of the participants’ attempt to resolve the dissonance between the two attitudes, which is associated with negative feelings. In order to minimize these negative feelings, participants were motivated to engage in a more thorough information processing and to examine relevant information. In another study of Goldstein and colleagues [30], IED positively predicted participants’ chocolate consumption even when implicit and explicit attitudes were unrelated to the behavior. It was suggested that due to the discrepancy, the focus on the object (chocolate) was intensified and thereby increased the occurrence of disinhibited eating. These findings demonstrate that implicit and explicit attitudes can be in conflict, which in turn impacts behavior. Moreover, Karpen and colleagues [32] revealed that the relationship between participant’s explicit attitudes towards alcoholic beverages and alcohol consumption was moderated by IED. More precisely, explicit attitudes were not a significant predictor for alcohol consumption when IED was strong but a significant predictor when IED was low.

Also in the context of physical activity, it has been shown that IED exists and that it impacts behavior [33, 34]. For example, the lower IED was in a sample of fitness club exercisers, the more successful they were in achieving their ideal exercise frequency [33]. In another study, discrepancy between explicit and implicit health measures regarding PA was negatively associated with the length to participate in a one year long exercise program [34]. These findings demonstrate that there is a direct link between IED and PA behavior. It is, however, unclear whether IED also acts as a moderator of the relationships between explicit attitude and physical activity (PA) (as it was the case in the study of Karpen et al. [32] regarding alcohol consumption) and explicit attitude and intention.

New insights into these effects can help to understand the way implicit and explicit attitudes jointly guide PA, and thereby provide input to improve interventions that are aiming to enhance people’s activity levels. PA behavior has been addressed by means of numerous health interventions [35], as increased activity is known to have significant health benefits [36]. Yet, around 23% of the global adult population [36] and 80% of the global adolescent population [36, 37] are not sufficiently active, thereby increasing their risk for the development of noncommunicable diseases, such as cardiovascular diseases or diabetes [36]. Therefore, more insight into additional influencing factors, such as the effect of IED, could be helpful. Thus far, research has found that social-cognitive determinants such as a more positive explicit attitude towards PA, stronger perceived norms (i.e. the perceived norm that one should be active), stronger modeling (i.e. perceiving significant others in one’s environment as active), and more self-efficacy (i.e. perceiving oneself as capable of performing the behavior even in difficult situations) lead to a higher intention to be physically active [38–42]. Although intention does not always result in the translation of behavior – a phenomenon called the intention-behavior gap – it is one of the most proximate determinants of behavior and vital in the process of initiating a behavior [43]. Also regarding PA, a higher intention is more likely to result in PA behavior [38, 44–46]. Moreover, a more positive explicit attitude towards PA does not only result in a higher intention but also in greater PA levels [5, 39, 47]. Studies concerning the impact of explicit cognitions mostly concern the effects of explicit attitude which have been found to explain around 30% of variance in PA intention [48]. Therefore, explicit attitudes have been classified as an important and central predictor for PA engagement [47–51] and it is recommended that interventions reinforce attitude change in order to facilitate PA engagement and adherence [52]. In recent studies, also implicit attitudes were shown to be associated with PA levels [9, 18, 53, 54]. For example, exercisers hold more positive automatic associations towards PA than non-exercisers [53] and implicit attitudes predict PA behavior above and beyond the aforementioned social-cognitive determinants [9]. Moreover, a former study showed that implicit attitudes moderate the relationships between certain explicit cognitions (i.e. perceived cons, self-efficacy) and intention as well as between certain explicit cognitions (i.e. self-efficacy) and PA behavior [55]. The present study extends the previous study and adds new insights into the influence of IED on the relationship between explicit attitude and intention/PA behavior.

Until now, it is clear, that explicit attitudes play, besides other explicit cognitions (social norms, social modeling, self-efficacy) and implicit attitudes, a significant role in the prediction of PA. It remains unclear however, whether explicit attitudes are still strongly associated with PA behavior when explicit attitudes are discrepant from the implicit attitude (which is also associated with PA). Karpen et al. [32] demonstrated that high IED weakens the predictive power of explicit attitudes regarding behavior and argued that as a result of the discrepancy, the information regarding the target (behavior) are inconsistent. This in turn makes it harder for the individual to judge about and to move towards the target behavior. Based on this, we first explored whether IED is present in our sample and we expect it to be existent (Hypothesis 1). Secondly, we investigated whether the predictive power of explicit attitudes regarding PA *behavior* is also moderated by IED. We expected IED to moderate the relationship between explicit attitudes and PA behavior with explicit attitudes being a stronger predictor for PA behavior when IED is low and a weaker predictor for PA when IED is high (Hypothesis 2[H2]; Fig. 1).

**Fig. 1:** Does IED moderate the relationship between explicit attitude and PA behavior (H2) and the relationship between explicit attitude and PA intention (H3)?

According to social-cognitive models, explicit attitudes are strongly associated with *intention.* Intention does not always translate into actual behavior [43], however, it is the most proximal determinant for (PA) behavior [45, 56–58]. As high IED has shown to weaken the effect of explicit attitude on behavior [32], we argue that high IED should also weaken the effect of explicit attitude on intention. Hence, on top of the second hypothesis, we investigated whether IED also moderates the relationship between explicit attitude and *intention*. We expected that the relationship between explicit attitude and intention is moderated by IED with greater IED leading to a weaker relationship between explicit attitude and intention and lower IED leading to a stronger relationship between explicit attitude and intention (Hypothesis 3 [H3]; Fig. 1). Gaining insight into these effects could help to understand whether interventions aiming to increase PA intention and behavior by changing or fostering explicit attitudes have to take discrepant attitudes into account.

## Method

### Design

The study at hand is part of a larger study in which we investigated how implicit attitudes synergistically interact with explicit cognitions in the prediction of PA intention and behavior [55]. In the current study, the emphasis is on the moderating effect of IED. A three-wave longitudinal study was conducted with measurements at baseline (T0) and follow-ups after one month (T1) and after three months (T2).

### Ethical approval

Ethical approval for this study was obtained from the Medical Ethics Committee of Zuyderland (METC Z.), the Netherlands (15-N-169).

### Participants and recruitment

The study was conducted at the Behavioral and Experimental Economics Laboratory (BeeLab) of a Dutch University. The BeeLab holds a database of students who are willing to participate in experiments, which was used to recruit participants for this study. Most students in the database were German or Dutch native speakers and, therefore, the study was conducted in both these languages. If a student had indicated German or Dutch as mother tongue, then he or she was invited to participate via email. No further inclusion criteria needed to be met. At baseline, 1690 students were invited out of which 340 participated (i.e. 20% response rate). The low response rate could be explained by the fact that the subject pool is not updated regularly and thus also contains students who are finished with their studies. Also the requirement to come twice to the lab within a period of one month in order to receive one’s incentive might have been a barrier for participation. At T1, 240 students participated and after three months, 128 students took part.

### Procedure

All students who met the inclusion criteria of having German or Dutch as mother tongue received an invitation via email stating the subject of the study (i.e. physical activity and related cognitions). Further, students were informed about the three waves of measurement and that each measurement consisted of two tasks, which together took around 25 min to complete. Further, it was explained that there were no risks related to the participation and that all data would be gathered and analyzed anonymously. For the completion of the first two measurements, students received €15 and another €7.50 when having completed the third measurement. When willing to participate, students could choose their preferred timeslot on two given days. An e-mail reminder was sent one day before participating. On the day of participation, participants were welcomed in the lab, received instructions and provided written informed consent. To assess their implicit attitudes towards PA, they first completed a Single-Category Implicit Association Test (SC-IAT; Karpinski & Steinman, 2006) and subsequently filled in a questionnaire to obtain their explicit attitude. Since we know that PA intention and behavior are also strongly associated with social norms, social modeling and self-efficacy [38, 59], we assessed these constructs as well in order to be able to demonstrate the effect of IED on intention and behavior, independent of these other cognitions. The questionnaire had to be completed after the SC-IAT as it is expected that prior questions about PA would trigger related thoughts and could thereby affect the reaction time during the SC-IAT (Bargh et al. 2000). In the questionnaire, the following constructs were assessed in the following order: explicit attitude comprised of perceived pros and perceived cons, social norms and social modeling, self-efficacy, intention, and physical activity levels.

### Measurements

#### Implicit attitude assessment task

Implicit attitudes towards PA were assessed by using the SC-IAT which showed adequate internal reliability and predictive validity in previous studies [18, 60, 61]. Additionally, the SC-IAT was used in former studies in which it successfully predicted objectively-measured PA [9] as well as unintentional PA [9, 18].

In the computerized tasks, participants were asked to indicate as fast and accurately as possible whether presented stimuli belonged to one of two given categories. The task consisted of two blocks which contained 24 practice trials and 72 test trials. In one block ‘physical activity or negative’ built a category and ‘positive’ the other category. In the other block, categories were reversed, thus ‘physical activity or positive’ was one category and ‘negative the other. The underlying assumption is that the stronger an implicit association is, the faster the reaction. Hence, if a person has negative implicit associations with being physically active he or she would be quicker in categorizing the displayed stimuli when ‘physical activity or negative’ are one category than when ‘physical activity or positive’ build a category. To ensure that reaction times were not influenced by the order of the blocks, the order of the two blocks was counterbalanced. Thus some participants had the categories ‘physical activity or positive’ and ‘negative’ first and the reversed categories subsequently, whereas other participants had the block ‘physical activity or negative’ and ‘positive’ first and the reversed pattern afterwards. Throughout the whole SC-IAT, labels for the two categories were displayed on the left or right upper part of the screen. If the presented stimulus belonged to the category that was displayed on the left part of the screen, participants had to press *e* on their keyboard. When the stimulus belonged to the category that was presented on the right upper part of the screen, the participant had to press *i* on the keyboard. The words were presented in a random order and equally frequent. In case that an incorrect answer was given, a red X appeared on the screen until the participant corrected the answer as recommended by Greenwald et al. [62].

The selection procedure for the stimuli was as follows: based on their valence and arousal norms, positive and negative words were chosen from the Affective Norms for English Words (ANEW) [63]. Words representing PA were selected from the studies of Conroy et al. (2010) and Hyde et al. (2010) who also used the SC-IAT to measure implicit attitudes towards PA. All selected words were translated forth and back from English to Dutch and German by native speaking researchers of the University. The positive and negative words were then pretested regarding the perceived levels of valence (1 = very negative to 9 = very positive), arousal (1 = not arousing at all to 9 = very arousing), and familiarity (1 = very unfamiliar to 9 = very familiar). PA related words were pretested regarding their representativeness for PA (1 = not representative at all, 2 = not so strongly/a bit representative, 3 = strongly representative). The pre-test was done among 26 German and 22 Dutch native students of the University. *Love, freedom, joy, success*, and *party* were selected as positive words (translated from German and Dutch); *depression, demon, lie, infection*, and *poison* were selected as negative words (translated from German and Dutch). The seven words *running, biking, kickboxing, sprint, jogging, lifting weights*, and *sit-ups* were selected as words to represent PA (translated from German and Dutch).

By means of the Inquisit Millisecond 4.0 software [64], the SC-IAT was programmed and presented. The script was based on the manual of Karpinski and Steinman [60]. The implicit attitude was indicated by d-scores that were calculated by the software using the improved scoring algorithm as described by Greenwald et al. [62]. In this procedure, the average response time for the test block with the categories *physical activity or negative*/*positive* is subtracted from the average response time of the reversed test block, in this case *physical activity or positive*/*negative.* Afterwards, the score gets divided by the standard deviation of all correct response times of the test trials. Normally, d-scores range from − 2 to 2. Reaction times of our sample did not exceed this range. Positive scores indicate a positive implicit attitude and negative scores indicate a negative implicit attitude. The higher the score, the more positive the implicit attitude. Based on the procedure as described in Karpinski and Steinman (60) we assessed the internal reliability of the SC-IAT by dividing the SC-IAT into thirds (blocks of 24 test trials) and calculated a separate d-score for each third. A measure of internal consistency was obtained by calculating the average intercorrelation among these scores and applying the Spearman-Brown formula that revealed an acceptable value of *r* = .83. Test-retest correlation between d-scores at baseline and at T1 showed a significant moderate correlation of *r* = .43 (*p* < .001) and test-retest correlation between d-scores at T1 and at T2 showed a low correlation of *r* = .17 (*p* = 06). Latter result is comparable to the results of other studies, which demonstrated weak test-retest reliabilities for the SC-IAT regarding other topics [65] as well as in the context of PA [66].

#### Questionnaire

The questions to assess explicit cognitions were based on the I-Change model [46, 56], which was used in former studies to assess PA related cognitions [41, 42, 67]. The following definition of adequate PA was shown to the participants with the option to reread it at any time while answering the questionnaire: Being sufficiently active is defined as being moderately physically active five times a week for at least 30 min. Being moderately active means an increase in heart rate that is induced by activities such as brisk walking [68]. The full questionnaire can be found at 10.1186/s40359-018-0229-0.

Explicit attitude was assessed on a 5-point Likert Scale with two scales measuring *perceived pros* and *perceived cons*, each expressed by 10 statements. Pros were measured by affective items such as ‘Being adequately physically active is’ (1) ‘very enjoyable’ to (5) ‘not enjoyable’, and instrumental items such as ‘Being adequately physically active is’ (1) ‘very good for my health’ to (5) ‘not good for my health’. Items were reversed, so that higher items represent the perception of more advantages. Based on low factor loadings, three items from the pro scale were removed (Ω = .75). Perceived cons were measured by affective items such as ‘Being adequately physically active is’ (1) ‘very unpleasant’ to (5) ‘not unpleasant’, and instrumental items such as ‘Being adequately physically active is’ (1) ‘too expensive’ to (5) ‘not expensive’. Lower scores indicate the perception of fewer disadvantages. Three items were removed from the scale, also due to low factor loadings (Ω = .70). For the analysis, a sum score for the con scale and a sum score for the pro scale were created. Both scale scores were added to represent one scale score for explicit attitude (range 14–70) that was used in the analyses. The higher the score, the more positive the explicit attitude.

*Social norms* and *social modeling* were each assessed by four questions on a 5-point Likert scale. Whereas norm items assessed expectations of family members, partners, and friends, with respect to PA, modeling items assessed the PA behavior of those. An example for a social norm item is ‘My partner’ (1) ‘doesn’t expect me at all to be physically active’ to (5) ‘certainly expects me to be adequately physically active’. An example for a modeling item is ‘Most of my family members are adequately physically active’ with answers ranging from (1) ‘totally disagree’ to (5) ‘totally agree’. The mean score for norms was included in the analyses (Ω = .62). The higher the score, the stronger the norms. Factor saturation regarding social modelling was estimated as insufficient (Ω = .34), which was also demonstrated by low factor loadings. Hence, social modeling items were included separately in the analyses.

*Self-efficacy* was measured on a 5-point Likert scale. Nine statements asked participants to indicate to what extent they expect themselves to be able to be adequately physically active in different situations, for instance ‘I find it difficult/easy to be adequately physically active when I am very busy’ with answers ranging from (1) ‘very difficult’ to (5) ‘very easy’. Based on their low factor loadings and their content (i.e. items referring to a specific activity instead of physical activity in general), three items were removed and a mean scale score was created of the remaining six items and included in the analyses (Ω = .66). A higher score indicates higher levels of self-efficacy.

Three items measured a person’s *intention* to be adequately active. On a 5-point Likert scale the first item assessed whether respondents were planning to be adequately physically active within the next three months ranging from (1) ‘no, not at all’ to (5) ‘yes, absolutely’. The second item asked whether respondents were motivated to be adequately physically active within the next three months with answer options from (1) ‘totally disagree’ to (5) ‘totally agree’, and the third item assessed how high chances were to be adequately physically active within the next three months with answers ranging from (1) ‘very little’ to (5) ‘very high’. The mean score of all three items was included as scale score for intention in the analyses (Ω = .89) with higher scores representing a stronger intention.

*Physical activity levels* were assessed by using the Short Questionnaire to Asses Health-enhancing physical activity (SQUASH) [69]. The SQUASH has been used in former studies to assess PA [41, 42, 67] and the reliability and validity were demonstrated [69, 70]. The SQUASH assesses different activities (e.g. commuting activities, household activities, leisure time activities). For each activity the frequency, duration (in minutes), and intensity (light/moderate/intense expressed in metabolic equivalent values, METs) were assessed. Total minutes of an activity were calculated by multiplying the frequency of an activity by its duration. The total minutes in turn were multiplied by the respective intensity in order to get an activity score for each activity (Wendel-Vos et al., 2003). By the sum of all different activity scores, a total activity score was obtained. The higher the score, the more active a person is.

Further, age (‘How old are you?’) and gender (‘What is your gender?’) were assessed and included in the analyses. Also participants were asked whether they were unable to be currently physically active and in the recent past due to an illness (‘Do/did you suffer from an illness that makes/made it impossible for you to be physically active, e.g. brain bleeding or cancer?’). As none of the participants answered the question with ‘yes’, data of all participants were included.

##### Analyses

All analyses were done with SPSS version 23. In advance, differences between the German and Dutch versions of the tests were tested but not detected. In order to assess scale quality of the measurements used in the present study we calculated their dimensionality by means of exploratory factor analyses as well as McDonald’s omega as a less biased alternative to Cronbach’s alpha [71]. Based upon the sum of the squared loadings of items on the general factor. Omega_hierarchical_ estimates factor saturation and is used as an indicator of internal structure [72]. Values were calculated with the R program [73] and are displayed in the measurements section above.

To evaluate the effect of IED, an index was created by calculating the absolute value of the difference between the average of a participant’s standardized explicit attitude score and the standardized reaction times of the SC-IAT. This procedure is based on a number of previous studies on IED [19, 29, 74]. The index indicates where participants fall within the distribution of the sample on the explicit versus implicit measure, thus demonstrating the size of the discrepancy. When a person’s place in the distribution is the same on the explicit and implicit measure (e.g. low in the distribution on both measures, high in the distribution on both measures, and so on), the index has a value close to zero. The more the attitudes deviate from each other (e.g. low in the distribution of implicit attitudes and high in the distribution of explicit attitudes and vice versa), the higher the score on the index and the further away it is from zero. For an indication of the reliability of the IED index, we created three indices and conducted test-retest correlations between the indices that were created for the measurements at baseline and after one and three months. The baseline index showed a moderate correlation with the index after one month (r = .52, *p* < .001) and a weak correlation with the index after three months (r = .29, <.001).

For the second hypothesis and in order to assess cross-sectional and longitudinal effects of the moderating effect of IED on the relationship between explicit attitude and PA, three regressions were conducted. For short-term effects, we regressed participant’s PA levels at T0 on age and gender in step one, baseline explicit attitudes, social norms, social modeling, self-efficacy, implicit attitude, and IED in a second step, and added the interaction between IED and explicit attitude in a third step. To assess long-term effects, the same regression was repeated but with PA at T1 and T2 as dependent variable. When the interaction between explicit attitude and IED was significant, we conducted stratified analyses with IED.

To investigate the third hypothesis and short-term and long-term effects of IED on the relationship between explicit attitude and intention, we conducted three regressions each with intention at baseline, at T1 and at T2 as dependent variable. Baseline variables were again added in three steps of a regression. Age and gender in step one, explicit attitudes, social norms, social modeling, self-efficacy, implicit attitudes and IED in step two, and the IED by explicit attitude interaction in step three. Main effects of the regression analyses were interpreted in the second step of the regression and the two way interaction in the third step [75]. Cases with missing values were not included in the analyses.

## Results

### Characteristics of the sample

The mean age of the sample at baseline (*N* = 340) was 21 years (SD = 2.11) and 61% was female. Of the sample, 91% met the Dutch Guideline for physical activity, which was, at the time the study was conducted, to perform moderate or vigorous activities for at least 150 min per week [68]. After one month, 240 students participated (71% of baseline, 64% female, mean age = 21, SD = 2.12) and after three months, 128 students (38% of baseline, 69% female, mean age = 22, SD = 2.17) took part. At follow-up one and two, more men dropped out than women (T1: OR = 0.55. 95% CI [.04, 1.00]. *p* = .02; T2: OR = 0.51, 95% CI [.02, 1.00], *p* = .01). No other variables predicted dropout. We included gender, a significant predictor of dropout, in all further analyses.

### Associations between predictors

Descriptive statistics and correlations between the study variables at baseline are presented in Table 1. IED had a range of 0.00–4.29 (M = 1.06, SD = .81) and the mean differed significantly from zero (t = _(339)_ 24.27, *p* < .001). The distribution of IED scores at baseline is displayed in Fig. 2. IED was not correlated with any of the measured explicit cognitions. Explicit attitudes and implicit attitudes were significantly correlated with each other (r = .11). Also, explicit attitude was correlated with intention, self-efficacy, social modeling by family members, PA, and social modeling by colleagues. Implicit attitudes were not significantly correlated to any other explicit cognitions.

**Table 1:** Means, standard deviations and correlations between study variables at baseline

	M (SD)		Correlations								
		1	2	3	4.1	4.2	4.3	4.4	5	6	7
1. Explicit attitude	56.30 (6.22)										
2. Implicit attitude	.1160 (.3310)	.11*									
3. Social norms	3.89 (.74)	.07	.01								
4.1. Social modeling (partner)	3.48 (1.20)	.08	.06	.34**							
4.2. Social modeling (family members)	3.43 (1.13)	.26**	.01	.15**	.10						
4.3. Social modeling (friends)	3.55 (.91)	.12*	.07	.18**	.33**	.13*					
4.4. Social modeling (colleagues)	3.31 (.83)	.11*	.08	.15**	.15	.13*	.44**				
5. Self-efficacy	2.60 (.62)	.45**	.08	−.09	.12	.14*	.02	.03			
6. Intention	4.43 (.67)	.57**	.06	.08	.11	.21**	.24**	.19**	.40**		
7. Physical activity	4959.03 (3187.16)	.24**	.07	.02	.02	.06	.04	.02	.20**	.24**	
8. IED	1.06 (.81)	−0.10	.02	.04	−.005	−.05	.04	.06	−.04	−.10	.01

*p < .05

**p < .01

**Fig. 2:** Distribution of IED at baseline (N = 340)

#### Does IED moderate the relationship between explicit attitude and PA behavior (at T0, T1, and T2)?

The interaction between IED and explicit attitude was not significant for PA at T0 (β = −.004, *p* = .97, 95% CI [− 73.55, 76.45]) nor at T1 (β = −.03, *p* = .85, 95% CI [− 106.06, 87.96]) or at T2 (β = .04, *p* = .87, 95% CI ([− 124.42, 146.91]). PA at T0 was significantly associated with self-efficacy (β = .22, *p* = .02, 95% CI [132.39, 1622.10]) and IED (β = −.16, *p* = .05, 95% CI [− 1072.79, 8.78]), demonstrating that a higher IED is associated with lower PA levels.

At T1, PA was significantly associated with self-efficacy (β = .38, *p* < .001, 95% CI [706.49, 2668.20]) and with IED (β = −.20, *p* = .06, 95% CI ([− 1397.93, 40.93]), also indicating that a high IED is associated with less PA.

After three months, PA was again significantly related to self-efficacy (β = .43, *p* = .005, 95% CI [539.93, 2801.46]), but not with IED (β = −.17, *p* = .24, 95% CI [− 1470.75, 382.83]). The results for all predictor variables are displayed in Table 2.

**Table 2:** Coefficients of the hierarchical multiple regression analysis with PA at T0, T1, and T2 as dependent variable. Interaction of explicit attitude with IED is added in step 3

Block	Independent variables	PA at T0					PA at T1					PA at T2				
		B	SE	β	95% CI	p	B	SE	β	95% CI	p	B	SE	β	95% CI	p
1	Gender	261.57	418.49	.05	−565.38 - 1088.52	.53	345.95	577.82	.06	− 800.86 - 1492.77	.55	1205.14	766.50	.21	− 332.95 - 2743.23	.12
	Age	61.48	89.65	.06	− 115.67 - 238.63	.49	115.02	119.70	.10	− 122.55 - 352.59	.34	70.62	163.71	.06	−257.88 - 399.13	.67
2	Gender	735.93	439.89	.15	− 133.76 - 1605.63	.10	1034.48	598.19	.18	−154.30 - 2223.26	.09	1946.78	795.76	.35	341.98–3551.59	.02
	Age	101.06	90.78	.09	−78.42 - 280.53	.27	155.86	120.06	.13	−82.74 - 394.45	.20	309.18	166.63	.26	−26.87 - 645.22	.07
	Explicit attitude	25.49	41.02	.06	−55.61 - 106.59	.54	1.79	58.98	.00	−115.42 - 119.01	.98	−82.54	96.80	−.16	− 277.77 - 112.68	.40
	Social Norms	30.49	315.84	.01	− 593.94 - 654.93	.92	494.88	450.84	.12	− 401.06 - 1390.83	.28	− 260.58	585.46	−.06	− 1441.28 - 920.12	.66
	Social Modeling (partner)	−67.41	191.94	−.03	− 446.88 - 312.05	.73	−282.51	249.60	−.12	−778.55 - 213.52	.26	−121.58	296.57	−.05	− 719.66 - 476.51	.68
	Social Modeling (family members)	−48.50	184.96	−.02	− 414.17 - 317.18	.79	−75.17	258.80	−.03	− 589.48 - 439.14	.77	− 524.24	329.07	−.23	− 1187.87 - 139.39	.12
	Social Modeling (friends)	31.56	270.10	.01	− 502.45 - 565.56	.91	252.93	381.10	.08	−504.42 - 1010.28	.51	−229.16	559.43	−.07	− 1357.35 - 899.03	.68
	Social Modeling (colleagues)	− 284.54	279.14	−.09	− 836.41 - 267.33	.31	− 151.79	376.39	−.05	−899.78 - 596.20	.69	− 916.08	494.37	−.29	− 1913.08 - 80.92	.07
	Self-efficacy	877.24	376.75	.22	132.39–1622.10	.02	1687.35	493.56	.38	706.49–2668.20	<.001	1670.69	560.70	.43	539.93–2801.46	.005
	Implicit attitude	1224.04	690.54	.15	−141.20 - 2589.28	.08	1648.47	971.16	.18	− 281.52 - 3578.45	.09	1389.70	1271.89	.15	− 1175.31 - 3954.72	.28
	IED	− 532.00	273.53	−.16	−1072.79 - 8.78	.05	− 678.50	362.02	−.20	−1397.93 - 40.93	.06	−543.96	459.56	−.17	−1470.75 - 382.83	.24
3	Gender	738.39	446.12	.15	−143.67 - 1620.45	.10	1025.90	603.28	.18	− 173.19 - 2224.98	.09	1958.24	807.82	.35	327.99–3588.48	.02
	Age	101.07	91.10	.09	−79.06 - 281.20	.27	158.37	121.48	.13	−83.09 - 399.82	.20	307.55	168.83	.26	−33.16 - 648.26	.08
	Explicit attitude	24.69	46.14	.06	−66.53 - 115.92	.59	8.01	68.12	.02	− 127.39 - 143.41	.91	−90.42	108.65	−.17	− 309.68 - 128.85	.41
	Social Norms	30.32	317.01	.01	−596.46 - 657.10	.92	492.73	453.48	.12	− 408.61 - 1394.07	.28	−258.54	592.32	−.06	− 1453.89 - 936.82	.66
	Social Modeling (partner)	−67.10	192.80	−.03	− 448.29 - 314.10	.73	−284.98	251.34	−.12	− 784.54 - 214.58	.26	− 114.03	303.35	−.05	− 726.22 – 498.16	.71
	Social Modeling (family members)	−48.36	185.66	−.02	−415.44 - 318.71	.79	−76.97	260.41	−.03	− 594.57 - 440.63	.77	− 530.75	335.12	−.23	− 1207.05 - 145.55	.12
	Social Modeling (friends)	31.33	271.13	.01	−504.75 - 567.41	.91	254.33	383.28	.08	− 507.48 - 1016.13	.51	− 234.93	566.91	−.08	− 1378.99 - 909.14	.68
	Social Modeling (colleagues)	−284.09	280.38	−.09	− 838.46 - 270.28	.31	− 159.07	380.50	−.05	− 915.36 - 597.21	.68	− 907.00	502.99	−.29	− 1922.09 - 108.08	.08
	Self-efficacy	878.85	380.44	.22	126.66–1631.05	.02	1678.98	498.34	.38	688.48–2669.48	<.001	1675.05	567.75	.43	529.29–2820.81	<.001
	Implicit attitude	1239.85	807.07	.15	−355.87 - 2835.56	.13	1551.96	1106.57	.17	− 647.48 - 3751.39	.16	1521.38	1508.29	.16	− 1522.47 - 4565.23	.32
	IED	− 527.40	299.82	−.16	− 1120.19 - 65.40	.08	− 711.28	404.67	−.21	− 1515.61 - 93.05	.08	−500.30	533.12	−.15	− 1576.18 - 575.58	.35
	IED x Explicit attitude	1.45	37.93	.004	−73.55 - 76.45	.97	−9.05	48.81	−.03	−106.06 - 87.96	.85	11.24	67.22	.04	−124.42 - 146.91	.87

*Note.* B = unstandardized regression coefficient; β = standardized regression coefficient; SE = standard error; 95% CI = 95% confidence interval

### Post-hoc analyses

As a result of the null-findings, we conducted post-hoc analyses, in which we tested whether the relationship between the *affective* explicit attitude and PA is moderated by the discrepancy between the affective explicit attitude and the implicit attitude. This is based on the assumption that implicit attitudes are grounded in affective associations and therefore rather comparable to affective explicit attitudes than to instrumental explicit attitudes [33]. Hence, the question arises whether the discrepancy between these two constructs might influence the effect of the affective explicit attitude on PA behavior. We conducted the same three regression analyses as earlier, however instead of adding an overall explicit attitude score in step 2, we added affective explicit attitude and instrumental explicit attitude as single predictors, and instead of an index for the discrepancy between the overall explicit attitude (comprised of the affective *and* the instrumental dimension) and implicit attitudes, we added IED (affective) - an index for the difference between the implicit attitude and the affective explicit attitude only. In a third step, the interaction between IED (affective) and the affective explicit attitude was added. The other variables (e.g. self-efficacy, social norms) were added in the same steps as in the earlier regressions. PA at baseline and after one and three months served each as dependent variable.

At no measurement, the interaction between IED (affective) and the affective explicit attitude was significant (baseline: β = −.09, *p* = .43, 95% CI [− 227.14, 97.42]; T1: β = −.07, *p* = .62, 95% CI [− 257.33, 154.77]; T2: β = −.02, *p* = .94, 95% CI [− 318.27, 295.07]). At baseline and T1 however, IED (affective) was significantly associated with PA (baseline: β = −.19, *p* = .03, 95% CI [− 1136.26, − 54.08]; T1: β = −.24, *p* = .04, 95% CI [− 1556.51, − 41.76]), indicating that a greater discrepancy between the implicit attitude and the affective explicit attitude is associated with lower PA levels. The same pattern was found in the earlier analyses when IED was comprised of the discrepancy between both the affective *and* instrumental dimension of the explicit attitude and the implicit attitude.

Moreover, as IED was significantly associated with PA at baseline and T1, we tested whether the direction of the discrepancy plays a role in this regard or not. To do so, we conducted two additional regressions in which we added age and gender in step 1, explicit attitude, social norms, social modeling, self-efficacy, implicit attitude, and IED in step 2, and the direction of the dissonance (coded as dummy) as well as an interaction term between IED and the direction of the dissonance in step 3. For PA at baseline, the interaction term was not significant (β = 1.28, *p* = .10, 95% CI [− 1033.23, 11636.43]). For PA at T1, the interaction was significant (β = 2.55, *p* < .001, 95% CI [2698.91, 17946.37]) and additional simple slope analyses showed that IED was significant when the explicit attitude was higher/more positive than the implicit attitude (β = 1.76, *p* = .04, 95% CI [466.83, 12152.93]) but not vice-versa (β = −.51, *p* = .60, 95% CI [− 7058.48, 4158.91]).

#### Does IED moderate the relationship between explicit attitude and the intention to be active (at T0, T1, and T2)?

No significant interaction between IED and explicit attitude was found for intention at T0 (β = .03, *p* = .74, 95% CI [−.01, .02]). Explicit attitude (β = .43, p < .001, 95% CI [.03, .06]) and self-efficacy (β = .23, *p* = .007, 95% CI [.06, .39]) were significantly associated with T0 intention.

For intention at T1, the interaction between IED and explicit attitude was also not significant (β = .19, *p* = .17, 95% CI [−.01, .04]). Significant predictors were explicit attitude (β = .20, *p* = .05, 95% CI [.00, .85]), social modeling of family members (β = −.19, p = .05, 95% CI [−.22, .001]), and self-efficacy (β = .26, *p* = .01, 95% CI [.06, .48]).

At T2, explicit attitude (β = .58, *p* = .002, 95% CI [.02, .10]) and social modeling (partner) (β = .31, *p* = .02, 95% CI [.03, .25]) were significantly related to intention. The interaction between IED and explicit attitude was not significant (β = −.03, *p* = .89, 95% CI [−.03, .02]).

### Post-hoc analyses

As a result of the null-findings, we conducted post-hoc analyses, similar to the ones performed regarding question 1. This time we tested whether the relationship between the affective explicit attitude and intention is moderated by the discrepancy between the affective explicit attitude and the implicit attitude. This is based on the same reasoning that implicit attitudes are grounded in affective associations and therefore rather comparable to affective explicit attitudes [33]. The same regressions as earlier were conducted. Instead of an overall explicit attitude score, we added affective explicit attitude and instrumental explicit attitude as single predictors in step 2, and instead of an index for the discrepancy between the overall explicit attitude (comprised of the affective *and* the instrumental dimension) and implicit attitudes (IED), we added IED (affective) as an index for the difference between the implicit attitude and the affective explicit attitude. In a third step, the interaction between IED (affective) and the affective explicit attitude was added. The other variables (e.g. self-efficacy, social norms) were added in the same steps as in the earlier regressions. Intention at baseline and after one and three months served each as dependent variable.

At no measurement, the interaction between IED (affective) and the affective explicit attitude was significant (baseline: β = −.001, *p* = .99, 95% CI [−.04, .04]; T1: β = .15, *p* = .28, 95% CI [−.02, .07]; T2: β = −.13, *p* = .52, 95% CI [−.08, .04]). The same pattern was found in the earlier analyses when IED was comprised of the discrepancy between both the affective *and* instrumental dimension of the explicit attitude and the implicit attitude.

## Discussion

The current study is part of a larger study, which showed that explicit cognitions and implicit attitudes interact in the prediction of PA behavior and intention [55]. Previous studies have shown that explicit attitudes and implicit attitudes can be discrepant from each other (Brinol et al., 2006; Petty et al., 2006; Rydell and McConnell, 2006; Rydell et al., 2008; Goldstein et al., 2014; Maliszewski. 2011) and explicit attitudes can be a weaker predictor for behavior when this is the case [32]. The present study aimed to extend this idea with physical activity as target behavior, thereby adding new insights into two specific relationships and the role of IED in these relationships [55]. More precisely, we investigated the effect of IED on the influence of explicit attitudes on PA behavior as well as on intention.

IED was present but not very strong. Contrary to our hypotheses and former research [32] we did not find IED to moderate the relationship between explicit attitude on PA behavior at any of the three measurements. Although PA and explicit attitudes were correlated with each other (at baseline), explicit attitudes were not associated with PA behavior at any measurement point as demonstrated in the regression models. Therefore, it is logical that explicit attitudes regarding PA prediction were unaffected by discrepancy. Also IED did not moderate the relationship between explicit attitude and intention. The null-findings could be a result of the fact that IED was not very strong in the sample, which is reflected in the low mean and can also be seen in the distribution of IED (Fig. 2). This in turn could be due to the target behavior PA. The coherence between implicitly and explicitly measured attitudes regarding the same target is strong (as it was the case in the present study) when self-presentation concerns are weak and lower when self-presentation concerns are high [18, 76, 77]. Hence in the latter context, explicit attitudes are more likely to diverge from the unbiased (in terms of self-presentation) implicit attitudes. Karpen et al. [32] investigated the effect of IED regarding alcohol consumption, which is a socially more sensitive topic and strongly influenced by social desirability [78]. PA, on the other hand, is a much less socially sensitive topic, although also influenced by social desirability to some extent [79]. Therefore, implicit and explicit attitudes in the context of alcohol consumption are more likely to deviate strongly from each other (e.g. implicitly being in favor of alcohol consumption but as a result of social desirability indicating it explicitly as negative) that assumingly created a stronger dissonance, which in turn had a stronger effect on the predictive power of explicit attitudes. It should be taken into account however, that the extent of the true experienced dissonance in the present study is unclear as it was inferred from the discrepancy between scores. Therefore, asking participants whether they experienced dissonance-based discomfort or negative emotions, as it has been done elsewhere [29, 31], could be a valuable addition for future studies. Additionally, it should be noted that the evidence in support of the idea that social desirability results in IED is mixed [18, 76, 80]. According to Gawronksi [81] “the correspondence between implicit measures and self-reports is far more complex than just a matter of social desirability and self-presentation”(p. 144). Therefore, we encourage future studies to investigate possible other moderators of attitude congruence/dissonance, such as mindfulness (the ability to have insight into one’s inner processes) which has been identified as moderator in other domains [82], but not yet in health psychology.

Further, a post-hoc analysis revealed that the true score correlation between the perceived pros and perceived cons scale was rather low (−.47), indicating that a response bias, such as tendency to agree, might have been present when participants answered the questions on explicit attitude. Although we reversed the scores for perceived pros before adding perceived cons, thereby correcting for tendency to agree to some extent, this bias was possibly present. This could be another reason for the present null-findings. Further research working with explicit attitude should ensure to offer a balanced number of positively and negatively worded questions, also for other relevant constructs involved, in order to prevent this potential bias. To assess whether the discrepancy between the explicit attitude and the implicit attitude was low and did not show the anticipated effects as the explicit attitude was comprised of instrumental and affective dimensions, we conducted post-hoc analyses. In these analyses we created a discrepancy index between the implicit attitude and the affective dimension of the explicit attitude only. It is assumed that implicit attitudes are rather grounded in affective associations, which is somewhat comparable to affective explicit attitudes. It could be reasonable that the addition of the instrumental dimension to the index distorted the discrepancy between the rather similar constructs and also it’s possible effect. Post-hoc analyses however did not reveal any differences regarding the results.

### Additional finding

The study indicated that IED was negatively associated with baseline PA and PA behavior after one month. This finding applied to IED when it was comprised of the discrepancy between the instrumental and affective dimensions of the explicit attitude and the implicit attitude as well as when it was comprised of the discrepancy between the affective explicit attitude only and the implicit attitude. These findings are in line with studies demonstrating that IED affects (PA) behavior [19, 20, 29, 31, 33, 34]. The fact that IED was associated with PA behavior, even when explicit and implicit attitudes were not, is surprising but in accordance with the findings of Goldstein et al. [30]. IED predicted disinhibited eating while neither implicit nor explicit attitudes independently did. Contrary to Goldstein et al. [30] who found a stronger tendency for disinhibited eating with increasing IED and argued that dissonance intensified the focus towards the object, we found a negative relationship. Thus IED in the context of PA is rather detrimental as it was negatively associated with PA levels. This could be due to the fact that a person holds inconsistent information about PA, i.e. liking PA (explicitly) but feeling (implicitly) less positive about PA (as indicated by the post-hoc analyses), which makes it harder to move towards the behavior. Therefore, our results suggest that, when aiming for more PA engagement, one should take the congruence of attitudes into account even when attitudes themselves are not directly related to the behavior. However, in order to draw a more generalizable conclusion, follow-up studies are highly encouraged, especially because the sample of the current study was very active. It is possible that results in a less active sample might differ. For example, a less active sample might hold less favorable/stable explicit attitudes towards PA, which might weaken the relationship between explicit attitude and intention and thereby IED might be more influenceable. Also it would be valuable to investigate whether the effect of IED loses its effect on the long-term. In the present study IED did not affect behavior after three months anymore. This could either be due to the fact that individuals manage to dissolve the dissonance over time leaving the behavior unaffected or due to the lower power at the follow-ups.

### Limitations

When developing future studies, the following limitations of the study at hand could be taken into account. One limitation is that we only had students in our sample who on average had a quite positive explicit and implicit attitude towards PA, a high intention, as well as high activity levels. This is not representative for the general public [83] and could be another reason why dissonance was not as strong as expected. Therefore, future studies should make use of a sample with more varied attitudes towards PA. Also PA was measured by self-reports, which is likely to be inaccurate due to an over- or underestimation of activity levels [84]. The low correlations between PA and well-known predictors of PA, i.e. self-efficacy, intention, indicate a rather inaccurate measurement of PA. Despite the demonstrated validity of the questionnaire we used [69], it would be valuable to add objective measures such as accelerometers to provide an adequate report about PA levels [84, 85]. Moreover, positive and negative words used for the SC-IAT were unrelated to PA. This is a common approach, which has been used in various former studies regarding PA or other behaviors [17, 18, 30, 60, 61, 66]. It is possible, however, that implicit attitudes, and thereby IED, might have been different when negative or positive words related to PA (e.g. exhaustion or strength) were used. This would be in line with the assumption of the APE postulating that implicit attitudes are associative evaluations that “are best characterized as automatic affective reactions resulting from the particular associations that are activated automatically when one encounters a relevant stimulus” [13]. This is an avenue for further research. In addition, discrepancy was inferred from the index. Whether discrepancy was experienced by the population is rather unclear. Questions about the experience of discrepancy or associated negative feelings could be a valuable addition for future studies. Another way to assess discrepancy could be to measure participants’ automatic evaluations, share this information with them and let them rate eventual discrepancy between their reflective and automatic evaluation as it has been done by Brand et al. [33]. Also discrepancy was not manipulated, e.g. in an experimental setting. Therefore, causal inferences are rather hard to draw. In order to do so, follow-up studies with an experimental setting, such as performed in the study of Brand et al. [33], would be valuable. Lastly, the test-retest correlation between the indices was rather low, especially between the index at baseline and the index after three months, indicating that the instrumental is not stable over a longer period. It is unclear whether this is due to actual changes in IED, because of changes in measurement error due to time (also known as transient error), or an artefact of the substantial dropout over time.

## Conclusion

We did not find explicit attitudes to be a weaker predictor for PA behavior or intention when IED was high. However, this finding cannot automatically be transferred to other health behaviors. Instead, since findings regarding the effect of IED on behavior are inconsistent, it can be concluded that the relationship between attitude, attitude discrepancy, behavior, and intention is more complex and probably also determined by other variables, such as the type of behavior or a person’s ability to have insight into his or her implicit attitude or other inner processes (e.g. experiencing dissonance). Especially in the area of health psychology and health promotion, more research is needed in order to identify these behaviors and factors and how they interact with discrepant attitudes to eventually draw more generalizable conclusions.

## Data Availability

The datasets used and/or analyzed during the current study are available from the corresponding author on request.

## Abbreviations

BeeLab: Behavioral and experimental economics laboratory
IAT: Implicit Association Test
IED: Implicit-explicit discrepancy
MET: Metabolic equivalent of task
PA: Physical activity
SC-IAT: Single-Category Implicit Association Test
SQUASH: Short questionnaire to assess health-enhancing physical activity
T0: Baseline measure
T1: Follow-up after one month
T2: Follow-up after three months
